The article "Efficacy of Ginkgo biloba Extract Combined with Hormones in the Treatment of Sudden Deafness and Its Effect on the Reactivity of Peripheral Blood T Cell Subsets" was retracted in 2023. Reasons: signs of a paper mill; suspected computer-generated content; unreliable results or conclusions; concerns about the data.

# Efficacy of *Ginkgo biloba* Extract Combined with Hormones in the Treatment of Sudden Deafness and Its Effect on the Reactivity of Peripheral Blood T Cell Subsets

**DOI:** 10.1155/2022/2903808

**Published:** 2022-09-26

**Authors:** Zhenhua Zhu, Qi Wu, Ge Hu, Xianwen Wang, Wei Chang, Ji Bin, Weili Yang

**Affiliations:** Otolaryngology-Wide Head and Neck Surgery Department, The First Affiliated Hospital of Hunan University of Traditional Chinese Medicine, Changsha, 410007 Hunan, China

## Abstract

This work was aimed at exploring the efficacy of *Ginkgo biloba* extract combined with hormones in the treatment of sudden deafness and the influence on the reactivity of peripheral blood T cell subsets (PBTCSs). In this work, 64 patients with sudden deafness who were treated in The First Affiliated Hospital of Hunan University of Traditional Chinese Medicine from August 2019 to August 2022 were selected as the research objects. The patients were randomly divided into a hormone group (treatment with prednisone acetate, *n* = 34) and a combination group (treatment with Ginkgo-Damole combined with prednisone acetate, *n* = 30). After the two groups of patients were treated in different ways, their efficacy, symptom improvement, changes in blood rheology, and PBTCSs were compared. The total effective rates (TERs) of the hormone group and the combination group were 76.32% and 95.73%, respectively (*P* < 0.05). The fibrinogen contents of the patients in the combination group were obviously lower than those in the hormone group after 5 d, 7 d, and 10 d of treatment (*P* < 0.05). The high blood viscosity (HBV) values of patients in the combination group at 5 d, 7 d, and 10 d after treatment were greatly lower than those in the hormone group (*P* < 0.05). The low blood viscosity (LBV) values after 3 d, 7 d, and 10 d of treatment in the combined group were much lower in contrast to those in the hormone group (*P* < 0.05). The CD3+, CD4+, and CD4+/CD8+ in peripheral blood in the combination group were sharply higher while the CD8+ in the combined group was lower in contrast to the hormone group (*P* < 0.05). There was no visible difference in the incidence of adverse reactions between the two groups of patients after treatment (*P* > 0.05). In conclusion, the combined application of *Ginkgo biloba* extract and hormones could effectively improve the abnormal hemorheological indexes of patients with sudden deafness and effectively relieve the imbalance of PBTCSs, which was safe.

## 1. Introduction

Sudden deafness, also known as idiopathic deafness, refers to the sudden onset of unexplained sensorineural hearing loss within 72 hours [1]. In the process of diagnosis and treatment, it can be divided into low-frequency descending type, high-frequency descending type, flat descending type, and total deafness type. Different types of patients have different hearing loss and healing conditions [2]. Among them, the recovery rate of patients with low-frequency descending type can reach more than 75% after treatment, and the outcome is good; while the recovery rate of patients with total deafness is less than 20%, the outcome is poor and easy to relapse [3, 4]. At present, the research on the etiology and pathogenesis of sudden deafness has not yet reached a clear conclusion, and it is generally believed that it has a certain correlation with the blood supply disorder of the inner ear and the membranous labyrinth [5]. Studies have found that sudden deafness can be caused by viral or bacterial infections, or by certain obstacles in the human circulatory system [6]. In addition, it may be caused by immune system problems, some foreign pathogens invade the body, causing the body's balance to be disrupted and resulting in the occurrence of sudden deafness [7, 8]. Some patients may be accompanied by cold symptoms before the onset of sudden deafness, when the virus enters the inner ear, causing infection and inflammation, which may lead to hearing loss [6, 9]. Factors such as high mental stress, mood swings, irregular daily routines, and sleep disturbances may be the triggers for sudden deafness. The onset of the disease is acute, the overall treatment efficiency is low, and the efficacy is highly correlated with the onset time, so it is recommended to diagnose and treat within 1 week of onset [10, 11].

Sudden deafness is generally treated with drugs, including glucocorticoids (methylprednisolone or dexamethasone, etc.), *Ginkgo biloba* extract, nutritive nerve drugs and antioxidants, and fibrinogen-lowering drugs (lowering fibrinogen improves inner ear circulation) [12–14]. Glucocorticoids are more suitable for patients with various types of sudden deafness, exerting anti-inflammatory and antitumor effects, while *Ginkgo biloba* extract is suitable for improving blood circulation in the inner ear and reducing blood viscosity [15]. Studies have found that *Ginkgo biloba* extract has free radical scavenging effects, regulating effects on the circulatory system, and improving hemodynamics and tissue protection. Therefore, it plays a key role in the treatment of sudden deafness [16]. In addition, hyperbaric oxygen can be used as a rescue therapy for patients who have no obvious effect on conventional drug therapy [17].

However, the long-term use of glucocorticoids will affect the metabolism of sugar and fat in the body, causing problems such as hyperglycemia and hyperlipidemia, so it is necessary to strictly follow the doctor's guidance for medication [18]. In addition, patients with underlying diseases such as diabetes and hypertension need regular monitoring during medication and should choose a reasonable and safe medication strategy under the guidance of doctors [19, 20]. At present, a large number of studies have found that both glucocorticoids and *Ginkgo biloba* extracts have obvious curative effects on sudden deafness, but few studies have combined the two drugs, and the safety and efficacy of the combined use are still unclear. Some studies suggest that the occurrence of sudden deafness may be related to the immune status of the body [21]. However, whether it is possible to predict the efficacy of hormone combined with *Ginkgo biloba* extract in the treatment of patients with sudden deafness and the correlation between the two can be determined by detecting the level of T cell subsets in patients' peripheral blood. Therefore, this work selected patients with sudden deafness as the research object for analysis and discussion.

## 2. Materials and Methods

### 2.1. Research Objects and Their Grouping

64 patients with sudden deafness (sudden deafness within 72 hours, unexplained sensorineural hearing loss, and hearing loss in at least two adjacent frequencies ≥20 dBHL) who visited The First Affiliated Hospital of Hunan University of Traditional Chinese Medicine from August 2019 to August 2022 as the research objects. Among them, there were 27 male patients and 37 female patients, aged 20 to 85 years old, with an average age of 34.72 ± 12.15 years old. Patients were randomized into a hormone group (treated with prednisone acetate, *n* = 34) and a combination group (treated with Ginkgo-Damole combined with prednisone acetate, *n* = 30). The experiment was approved by the Medical Ethics Committee of The First Affiliated Hospital of Hunan University of Traditional Chinese Medicine, and the patients and their families understood the research content and methods and agreed to sign the corresponding informed consents.

Patients included had to satisfy the following items: (1) the initial visit time was 1 to 5 days after the onset of the disease; (2) the age was 20 to 85 years old; (3) the patients with normal blood pressure, liver and kidney function, blood sugar, blood lipids, and normal blood routine; and (4) patients who were willing to actively cooperate with treatment.

If any of the following conditions was satisfied, the patient had to be excluded: (1) poor general condition and unable to tolerate hormone therapy; (2) pregnant or breastfeeding women or allergic to treatment drugs; (3) cognitive impairment and unable to complete the hearing test; (4) allergic rhinitis and autoimmune diseases; and (5) hepatitis B and hepatitis C virus carriers and those with a history of immune diseases.

### 2.2. Research Methods

The included patients were divided into a hormone group and a combination group. The patients in the hormone group were treated with prednisone acetate. After getting up in the morning, the patient was required to take 60 mg of prednisone acetate (Guoyao Zhunzi H62020285, Gansu Fuzheng Pharmaceutical, 5 mg/tablet) orally 1 time/day. After 3 days of administration, it should reduce the drug dose, with prednisone acetate 30 mg/time and 1 time/day. The patients in the combination group were treated with Ginkgo-Damole combined with prednisone acetate. Ginkgo-Damole (Guoyao Zhunzi H52020032, Guizhou Yibai Pharmaceutical Co., Ltd., 10 mL added to 500 mL of 0.9% sodium chloride injection) was taken intravenously once a day. For combined treatment with prednisone acetate, the patients should take 60 mg of prednisone acetate (Guoyao Zhunzi H62020285, Gansu Fuzheng Pharmaceutical Co., 5 mg/tablet) orally after getting up in the morning once a day. After 3 days of administration, the dose was adjusted to 30 mg/time once/day. The two groups were treated continuously for 7 days as a course of treatment, and the curative effect was observed.  Figure 1 shows the structural formula of prednisone acetate.

### 2.3. Evaluation Standards

Symptoms improved: after the two groups of patients were treated in different ways, their symptoms (ear fullness, tinnitus, and vertigo) were scored for syndrome. The occurrence of the three symptoms was graded into 0 points (no symptoms), 2 points (mild ear fullness, tinnitus, and dizziness), 4 points (moderate ear fullness, tinnitus, and dizziness), and 6 points (severe ear fullness, tinnitus, and dizziness), respectively. It can calculate the degree of improvement of the patient's symptoms, the calculation method was

(1) $$\begin{array}{c} I={\text{Score}}_{T_{0}}-{\text{Score}}_{T_{1}}. \end{array}$$

In the above equation, *I* denoted the symptom improvement degree; Score_*T*_0__ refers to the syndrome score before treatment; and Score_*T*_1__ represents the syndrome score after treatment.

The therapeutic effect was assessed into cured, markedly effective, effective, and ineffective. Recovery: tinnitus and vertigo disappeared completely, and hearing returned to normal; markedly effective: tinnitus and vertigo disappeared, and hearing improved by more than 30 dB; effective: tinnitus and vertigo were relieved, and hearing was improved by 15-30 dB; and ineffective: tinnitus and vertigo were unchanged, and hearing was improved by less than 10 dB or even more serious. The calculation method of total effective rate (TER) was

(2) $$\begin{array}{c} \text{Total effective rate}=A+B+C. \end{array}$$

In the equation above, *A* represented the cure rate; *B* represented the markedly effective rate; and *C* represented the effective rate.

It should monitor and record the changes of hemorheology indexes and endothelial function indicators before treatment, 3 d, 5 d, 7 d, and 10 d after treatment. These indicators included fibrinogen, high blood viscosity (HBV), low blood viscosity (LBV), soluble vascular cell adhesion molecule-1 (sVCM-1), endothelin-1 (ET-1), and PBTCS indicators (CD3+, CD4+, CD8+, and CD4+/CD8+). The levels of sVCM-1 and ET-1 were detected by enzyme-linked immunosorbent assay (ELISA), and the detection kits were purchased from Shanghai Keaibo Biotechnology Co., Ltd. Detection of T cell subset levels: the whole blood samples were detected by EPICSX flow cytometer (Beckman-Coulter, USA). Fibrinogen, whole blood HBV, and LBV were detected by LG-R-80 type hemorheometer (Beijing Zhongqin Shidi Company).

### 2.4. Statistical Methods

Data processing in this work was performed using SPSS 24.0. Measurement data were expressed as the mean ± standard deviation ($\bar{x}\pm s$), the comparison within the group before and after treatment was performed by the Paired *t*-test, and the comparison between the two groups was performed by the Independent *t*-test. The enumeration data were expressed as percentage (%), and the pairwise comparison was made by variance analysis. To evaluate the correlation of PBTCSs with the pathogenesis of sudden deafness and its impact on the recovery of prognosis and the correlation was expressed by OR value (95% CI). The difference was statistically significant at *P* < 0.05.

## 3. Results

### 3.1. Basic Data of Patients

All patients included were divided into two groups and then treated with hormones (prednisone acetate) and Ginkgo-Damole combined with prednisone acetate. In order to analyze the curative effect of the two groups of patients after treatment in different ways, the basic information such as age and gender of the patients were first compared, and the results are shown in Table 1. It can be seen that the proportion of male patients in the hormone group and the combination group was 19.05% and 17.46%, respectively, and there was no visible difference (*P* > 0.05). The mean age and disease course of patients between the hormone group and the combination group showed no obvious difference (*P* > 0.05). In addition, the proportions of patients with different degrees of deafness, different tinnitus conditions, and symptoms in the two groups were compared, and the results are shown in Figure 2. The proportions of patients with moderate deafness, severe deafness, and total deafness in the hormone group were 21.23%, 49.56%, and 29.21%, respectively; while those in the combination group were 20.62%, 51.05%, and 28.33%, respectively. The proportions of patients with low-key tinnitus, high-profile tinnitus, and no tinnitus in the hormone group were 28.31%, 47.33%, and 24.36%, respectively; while those in the combination group were 28.06%, 49.08%, and 22.86%, respectively. The proportion of patients with ear fullness symptoms in the two groups were 52.33% and 50.47%, respectively; the proportions of patients with facial discomfort symptoms were 48.65% and 46.12%, respectively; and the proportions of patients with vertigo symptoms were 10.18% and 12.33%, respectively. The proportion of patients with different degrees of deafness, tinnitus, and accompanying symptoms showed no visible difference between two groups (*P* > 0.05).

### 3.2. Patient Efficacy and Symptom Improvement

The improvement of ear fullness, tinnitus, and dizziness was evaluated in the two groups of patients after treatment in different ways. The curative effect of patients was judged by four grades as cured, markedly effective, effective, and ineffective, and TER was calculated. The results are shown in Figure 3. In the hormone group, the patients with curative effect as cured, markedly effective, effective, and ineffective were 8 cases, 7 cases, 11 cases, and 8 cases, respectively. In the combination group, 11, 13, 3, and 3 patients were cured, markedly effective, effective, and ineffective, respectively. The number of cured and markedly effective patients was significantly higher in the combination group. The TER of the hormone group and the combination group were 76.32% and 95.73%, respectively, showing statistically great difference (*P* < 0.05). The improvement degrees of ear fullness, tinnitus, and dizziness in the hormone group patients were 1.52, 1.65, and 1.8, respectively; while those in the combination group were 2.31, 2.53, and 2.66, respectively, showing great difference statistically (*P* < 0.05).

### 3.3. Changes in Hemorheological Indexes of Patients

The two groups of patients were treated in different ways, and the changes of hemorheology indexes were monitored and recorded before treatment and after 3 d, 5 d, 7 d, and 10 d after treatment. The differences between the two groups at different times were compared; the results are shown in Figure 4.  Figure 4(a) showed the changes of fibrinogen. With the prolongation of treatment time, the fibrinogen content of the two groups of patients gradually decreased, and the fibrinogen content of the combination group decreased more obviously. No obvious difference in fibrinogen content was found before treatment and 3 days after treatment (*P* > 0.05). The fibrinogen contents of patients in the combination group at 5 d, 7 d, and 10 d after treatment were 3.19 ± 0.87 g/L, 2.89 ± 0.61 g/L, and 2.51 ± 0.83 g/L, respectively, which were lower than those in the hormone group (3.9 ± 0.64 g/L, 3.89 ± 0.54 g/L, and 3.55 ± 0.78 g/L, respectively); in addition, the fibrinogen contents of both groups were obviously lower than the contents before treatment (*P* < 0.05).  Figure 4(b) shows the changes of HBV. It suggested that with the prolongation of treatment time, HBV in both groups gradually decreased, and the decrease in HBV in the combination group was more obvious. HBV before treatment and 3 days after treatment showed no obvious difference (*P* > 0.05). The HBV levels of patients in the combination group at 5 d, 7 d, and 10 d after treatment (4.02 ± 0.6 mPa∗s, 3.98 ± 0.66 mPa∗s, and 3.66 ± 0.6 mPa∗s) were significantly lower than those in the hormone group (6.43 ± 0.55 mPa∗s, 5.89 ± 0.69 mPa∗s, and 5.72 ± 0.48 mPa∗s), and all were much lower than the levels before treatment (*P* < 0.05).  Figure 4(c) shows the changes of LBV. It indicated that with the prolongation of treatment time, the LBV of the two groups of patients decreased gradually, and the LBV of the combination group decreased more obviously, but the difference in between the two groups before treatment was not obvious (*P* > 0.05). The LBV of patients in the combination group at 3 d, 7 d, and 10 d after treatment (10.06 ± 0.49 mPa∗s, 7.35 ± 0.62 mPa∗s, and 6.48 ± 0.72 mPa∗s) were sharply lower compared to those in the hormone group (11.54 ± 0.65 mPa∗s, 9.37 ± 0.73 mPa∗s, and 8.79 ± 0.49 mPa∗s), and all were lower than the levels before treatment (*P* < 0.05).

### 3.4. Changes of Endothelial Function Indexes in Patients

The two groups of patients were treated in different ways, and the changes of endothelial function indexes were monitored and recorded before treatment and after 3 d, 5 d, 7 d, and 10 d after treatment. The differences between the two groups at different times were compared; the results are illustrated in Figure 5. Among them, Figure 5(a) revealed the changes of sVCM-1. With the prolongation of treatment time, the levels of sVCM-1 in the two groups were gradually decreased, and the levels of sVCM-1 in the combination group decreased more obviously. The sVCM-1 showed no great difference between the two groups before treatment and 3 days after treatment (*P* > 0.05). The levels of sVCM-1 in patients in the combination group were 203.54 ± 19.38 g/L, 185.43 ± 15.01 g/L, and 170.52 ± 19.02 g/L after treatment for 5 d, 7 d, and 10 d, respectively, which were notably lower than those in the hormone group (240.44 ± 19.92 g/L, 238.91 ± 20.45 g/L, and 236.88 ± 18.3 g/L), and all decreased than those before treatment (*P* < 0.05).  Figure 5(b) suggests the changes of Endothelin-1 (ET-1). As it illustrates the prolongation of treatment time, the levels of ET-1 in the two groups gradually decreased, and the levels of ET-1 in the combination group decreased more obviously. There was no obvious difference before treatment and 3 days after treatment (*P* > 0.05). The levels of ET-1 in the combination group at 5 d, 7 d, and 10 d after treatment (125.36 ± 17.81 g/L, 100.03 ± 19.4 g/L, and 85.93 ± 18.82 g/L) were notably lower than those in the hormone group (139.81 ± 18.15 g/L, 125.44 ± 20.59 g/L, and 118.92 ± 19.7 g/L), and all were effectively lower than those before treatment (*P* < 0.05).

### 3.5. Comparison of PBTCSs of Patients

Figure 6 demonstrates the comparison results of PBTCSs indicators of patients. No visible difference was found in CD3+, CD4+, CD8+, and CD4+/CD8+ between the hormone group and the combination group before treatment (*P* > 0.05). After different treatments, the CD3+, CD4+, and CD4+/CD8+ in the combination group were much higher in contrast to those in the hormone group (*P* < 0.05). The CD8+ in peripheral blood in the combination group was observably lower than that in the hormone group (*P* < 0.05).

### 3.6. The Incidence of Adverse Reactions

Figure 7 reveales the occurrence of adverse reactions (nausea, dizziness, skin allergy, and other adverse reactions) in the hormone group and the combination group patients after prednisone acetate and Ginkgo-Damole combined with prednisone acetate treatment, respectively. The proportions of patients with nausea, dizziness, skin allergy, and other adverse reactions in the hormone group were 8.21%, 11.37%, 5.34%, and 6.31%, respectively; while those in the combination group were 8.66%, 10.96%, 5.45% and 6.54%, respectively (*P* > 0.05).

## 4. Discussion

Sudden deafness is a sudden onset of sensorineural hearing loss manifested as unilateral hearing loss, which can be accompanied by tinnitus, ear blockage, dizziness, nausea, and vomiting. It usually occurs suddenly within 72 hours, and the hearing loss of two adjacent frequencies can be found to be greater than or equal to 20 dBHL during pure tone audiometry [22]. The causes of sudden deafness are more complicated and may be related to factors such as inner ear blood supply disorder and viral infection [23]. At present, the widely recognized virus infection theory, circulatory disorder theory, autoimmunity theory, and membrane labyrinth rupture theory are the main ones. The disease is more common in people with high blood pressure, arteriosclerosis, hypothyroidism, and low blood pressure [24]. According to the frequency and degree of hearing loss, it can be divided into: high-frequency descending type, low-frequency descending type, flat descending type, and total deafness type (including profound deafness). Low-frequency descending type: hearing loss at frequencies below 1,000 Hz (inclusive), at least 250 Hz and 500 Hz hearing loss ≥20 dBHL; high-frequency descending type: hearing loss at frequencies above 2,000 Hz (inclusive), at least 4,000 Hz and 8,000 Hz hearing loss ≥20 dBHL; flat descending type: hearing loss at all frequencies, 250-8,000 Hz average hearing threshold ≤80 dBHL; and totally deafness type: hearing loss at all frequencies, with an average hearing threshold of 250-8,000 Hz ≥81 dBHL [25]. Different types have different treatment options. Sudden deafness should be treated with glucocorticoid drugs and neurotrophic drugs in accordance with the doctor's order. Common drugs include prednisone and methylcobalamin. Treatment options include microcirculation-improving drugs (such as *Ginkgo biloba* extract) combined with glucocorticoids; ion channel blockers (such as lidocaine) are better for reducing high-profile tinnitus; and neurotrophic drugs (such as methylcobalamin). The research of Singh et al. [26] showed that if the drug treatment was not effective, hyperbaric oxygen therapy and stellate ganglion block therapy can also be given. With appropriate treatment, the patient's hearing can be gradually restored.

Currently, *Ginkgo biloba* extract is the most commonly used drug for the treatment of sudden deafness clinically. *Ginkgo biloba* extract is made from *Ginkgo biloba* leaves and extracted with appropriate solvents. The main component is *Ginkgo biloba* flavonoid glycosides. Its main function is that of ginkgo flavone glycosides, and the main functions include: (1) scavenging of free radicals: *Ginkgo biloba* extract removes excess free radicals in the body and inhibits lipid peroxidation in cell membranes; thereby, protecting cell membranes and preventing a series of damage to the cochlea caused by free radicals. (2) Adjustment to the circulatory system: arterial relaxation is produced by stimulating the release of catecholamines and inhibiting degradation, stimulating the production of prostacyclin and endothelial relaxation factor, and jointly maintaining the tension of arterial and venous blood vessels. (3) Hemodynamic improvement effect: the onset of sudden deafness is generally considered to be related to thrombosis, especially the blood vessels of the cochlea are slender peripheral blood vessels. Research by Suzuki et al. [27] found that *Ginkgo biloba* extract can reduce the viscosity of whole blood, increase the plasticity of red blood cells and white blood cells, and improve the blood circulation of the cochlea. (4) Tissue protection: *Ginkgo biloba* extract has a protective effect on body tissues, which can increase the supply of oxygen and glucose to ischemic tissues (including the cochlea).

In this work, patients with sudden deafness were selected as the research objects, and their therapeutic effects were investigated after prednisone acetate and Ginkgo-Damole combined with prednisone acetate, respectively. The results showed that with the prolongation of treatment time, the blood rheology indexes of fibrinogen content, HBV, and LBV in the two groups were gradually decreased, and the content of the combination group decreased more obviously. The fibrinogen content, whole blood HBV, and LBV of patients in the combined group were significantly lower than those in the hormone group at 5 d, 7 d, and 10 d after treatment, and were significantly lower than those before treatment (*P* < 0.05). This result is similar to the research result of Övet et al. [28], which may be due to the flavonoid glycosides in *Ginkgo biloba* extract exerting the effect of scavenging free radicals and protecting brain tissue. Ginkgolide can balance lipid peroxidation, increase the tolerance of cells to hypoxia, change blood rheology, and increase the plasticity of whole blood. After different treatments, the peripheral blood CD3+, CD4+, CD4+/CD8+ in the combined group were significantly higher than those in the hormone group, and the differences were statistically significant (*P* < 0.05). In addition, the peripheral blood CD8+ in the combined group was significantly lower than that in the hormone group, and the difference was statistically significant (*P* < 0.05). Such results are similar to the research results of Suzuki et al. [29]. It indicates that T cell subsets may have a certain correlation with the prognosis and efficacy of patients with sudden deafness. Patients with sudden deafness may have an imbalance of peripheral blood T cell subsets, and the combined treatment of *Ginkgo biloba* extract and hormones has a certain improvement effect on the imbalance of PBTCSs. No great difference was found in nausea, dizziness, skin allergy, and other incidence of adverse reactions between the hormone group and the combination group after different treatments (*P* > 0.05). It indicates that the treatment method of this study has certain safety for sudden deafness treatment.

## 5. Conclusions

In this work, patients with sudden deafness were included, two methods of prednisone acetate and Ginkgo-Damole combined with prednisone acetate were used to intervene, and the comprehensive efficacy of the two groups of patients was compared. The results showed that the combined application of *Ginkgo biloba* extract and hormones can effectively improve the abnormal hemorheological indexes of patients with sudden deafness and effectively relieve the imbalance of PBTCSs, showing high safety. However, the sample size included in this work was small and the sources were concentrated, so it may have a certain impact on the reliability of the research results. In addition, according to the results of this work, *Ginkgo biloba* extract combined with hormones had a good therapeutic effect on sudden deafness, but the mechanism of its effect was still unclear. Therefore, the above aspects needed to be improved and optimized in the follow-up research, so as to make the research more perfect.

## Figures and Tables

**Figure 1:** The structural formula of prednisone acetate.

**Figure 2:** The degree and symptoms of deafness in patients. Note: (a) showed the degree of deafness of the two groups of patients, where (A)–(C) represented moderate deafness, severe deafness, and total deafness, respectively; (b) showed the patient's tinnitus status, where (A)–(C) represented low-key tinnitus, high-key tinnitus, and no tinnitus, respectively; (c) represented other symptoms of the patient, where (A)–(C) represented ear fullness, facial discomfort, and dizziness, respectively.

**Figure 3:** Curative effect and symptom improvement. Note: (a) showed the comparison of the two groups of patients whose curative effects were, respectively, cured, markedly effective, effective, and ineffective; (b) showed the TER; and (c) showed the degree of improvement of the patient's symptoms, where (A)–(C) indicated ear fullness, tinnitus, and dizziness, respectively; ∗ indicated *P* < 0.05 compared with the hormone group.

**Figure 4:** Changes of hemorheological indexes in patients. Note: (a)–(c) showed the fibrinogen content, HBV level, and LBV level, respectively; ∗ indicated *P* < 0.05 to the hormone group; # indicated *P* < 0.05 compared with before treatment.

**Figure 5:** Changes of endothelial function indexes in patients. Note: (a) and (b) compared the sVCM-1 and ET-1, respectively; ∗ and # indicated *P* < 0.05 to the hormone group and the combination group before treatment, respectively.

**Figure 6:** Comparison of PBTCSs of patients. Note: (a): CD3+; (b): CD4+; and (c): CD8+; D: CD4+/CD8+; ∗ indicated *P* < 0.05 to the hormone group.

**Figure 7:** The incidence of adverse reactions. Note: (a)–(d) represented nausea, dizziness, skin allergy, and other adverse reactions, respectively.

**Table 1:** Basic data of patients.

Item	Type	Proportion (%)	
		Hormone group (*n* = 34)	Combination group (*n* = 30)
Gender	Males	12 (19.05%)	11 (17.46%)
	Females	9 (14.29%)	10 (15.87%)

Age (years old)		33.68 ± 10.98	35.08 ± 12.24

Disease course (h)		8.09 ± 2.55	8.21 ± 1.08

## Data Availability

The data used to support the findings of this study are available from the corresponding author upon request.
